# TAB2 Promotes the Biological Functions of Head and Neck Squamous Cell Carcinoma Cells via EMT and PI3K Pathway

**DOI:** 10.1155/2022/1217918

**Published:** 2022-08-08

**Authors:** Huijuan Liu, Hui Zhang, Haidong Fan, Su Tang, Junquan Weng

**Affiliations:** ^1^Department of Stomatology, Shenzhen People's Hospital (The Second Clinical Medical College, Jinan University, The First Affiliated Hospital, Southern University of Science and Technology), Shenzhen, 518020 Guangdong, China; ^2^Department of Stomatology, Pingshan District People's Hospital of Shenzhen, Shenzhen, Guangdong 518118, China

## Abstract

**Background:**

Transforming growth factor *β*_1_-activated kinase 1 binding protein 2 (TAB2) mediates a variety of biological processes through activated nuclear factor *κ*-light-chain-enhancer of activated B cell (NF-*κ*B) signaling pathways. TAB2 has been reported to be upregulated in a variety of tumors. However, little is known about its potential role in oral squamous cell carcinoma (OSCC). *Material and Methods*. Patients' clinicopathological and transcription data were obtained from The Cancer Genome Atlas (TCGA) database. Immunohistochemistry staining was used to determine TAB2 expression in OSCC tissues (IHC). The expression of TAB2 in OSCC cell lines was detected by western blotting. The CCK-8 test and flow cytometry assay were utilized to evaluate cell proliferation, apoptosis, and cell cycle in OSCC cell lines. Enrichment analysis and identification of predicted signaling pathways were performed by Gene Ontology and KEGG analysis. Finally, the expression of downstream signal molecules was performed using western blotting to validate the mechanism investigations.

**Results:**

TAB2 expression level was aberrantly upregulated in OSCC patients. TAB2 expression was shown to be inversely associated to prognosis. The phenotypic of OSCC cells was considerably impacted by TAB2. OSCC cells with deleted TAB2 exhibit decreased proliferation and increased apoptosis. Additionally, OSCC progression is aided by TAB2 overexpression. Further mechanism studies showed that TAB2 could regulate the progression of OSCC by mediating the upregulation of EMT and PI3K-AKT signaling pathways.

**Conclusion:**

This study sheds light on the carcinogenic role of TAB2 in OSCC and provides a potential therapeutic strategy.

## 1. Introduction

Oral squamous cell carcinoma (OSCC) is one of the leading global problems because of its most adverse effects on patients' life quality [1, 2]. This disease was characterized by high recurrence rate, cervical lymph node metastasis, and poor clinical outcome. Recent work suggests that human papillomavirus (HPV, primarily HPV-16) is an etiological cause of OSCC [3, 4] and tobacco and excessive alcohol are the main causes for its high incidence [5, 6]. Approximately 500,000 OSCC cases were diagnosed per year [2]. With remarkable improvement in the current standard multimodality therapies during recent years, the prognosis of OSCC remains poor. Recurrence and metastasis risk cause an undesirable 5-year overall survival rate, which varies between 30% and 50% [7, 8].

Numerous research conducted in recent years have shown that OSCC displays abnormal oncogenic protein expression and/or signaling pathway activation. For instance, epidermal growth factor receptor (EGFR) is overexpressed in 80–90% of OSCC tumors [9–11], and its high expression is correlated with poor progression-free survival and overall survival (OS). The cytokine interleukin-6 (IL-6) overexpression and its receptor are also contributing to a bad prognosis in OSCC [12]. As a very crucial part of the molecular mechanism, OSCC tumor formation is driven not only by the accumulation of genetic alterations but also by epigenetic changes [13, 14]. Histone modifications, noncoding RNA activity, DNA methylation, and RNA methylation are among epigenetic changes related to OSCC development [15, 16]. As an illustration, both in vitro and in vivo tumor growth is inhibited by silencing of the m6A demethylase alkB homolog 5 RNA demethylase (ALKBH5) [17, 18]. By increasing snail family transcriptional repressor 1 (SNAIL1) mRNA translation, the protein methyltransferase methyltransferase-like 13 (METTL13) promotes OSCC development and maintenance [19]. Therefore, it is necessary to elucidate the potential mechanism of oncogenesis and progression of OSCC.

Transforming growth factor *β*_1_-activated kinase 1 binding protein 2 (TAB2), an important component of the complex, serves as an adaptor that links mitogen-activated protein kinase 7 (MAP3K7) and TNF receptor-associated factor 6 (TRAF6) [20]. More pervasively, binding with TAB2 will promote cardiovascular development and maintain extracellular matrix (ECM) homeostasis [21, 22]. It has been reported to participate in activating transcription factor NF-*κ*B signaling pathway, which makes it contribute to the initiation of epithelial ovarian cancer [23]. Moreover, TAB2 functions as a mediator of drug resistance and might be a potential new target for reversing drug resistance and enhancing antiestrogen effects in breast cancer [24]. To date, there are no researches focus on the relationship between TAB2 and OSCC. Thus, the underlying molecular role of TAB2 in OSCC still needs to be revealed.

## 2. Results

### 2.1. TAB2 Expression Was Correlated with OSCC

To investigate whether TAB2 plays an important role in OSCC, *TAB2* mRNA expression was compared between HNSCC tissues and normal tissues according to the TCGA database. TCGA data revealed that *TAB2* were distinctively upregulated in tumor tissues (Figure 1(a)). Furthermore, TAB2 expression differed by clinicopathological parameters: TAB2 upregulated with tumor grade 4 compared with lower tumor grade (Figure 1(b)). Consistently, TAB2 expression changes were confirmed by our patients' cohort, and its protein expression was increased in OSCC samples as compared with paracarcinoma tissues (Figures 1(c) and 1(d)). Next, the effects of TAB2 on overall survival (OS) of OSCC patients were analyzed. The OS of TAB2 high expression group was shown to be shorter than that in the TAB2 low expression group (Figure 1(e)), indicating that TAB2 serves as a risk factor in OSCC. Therefore, our data showed that the upregulated level of TAB2 was correlated with OSCC.

### 2.2. Decrease in TAB2 Expression Inhibited OSCC Growth and Promoted Apoptosis

Oncogenes are often involved in tumor cell activities such as continuous proliferation, avoidance of growth inhibition, and resistance to apoptosis [25–27]. To investigate the function of TAB2 as a potential oncogene in OSCC cells, 6 HNSCC cell lines were selected and compared their TAB2 protein level (Figure 2(a)). Data showed that two OSCC cell lines (SCC4 and SCC9) present higher expression and one (SCC1) presents lower level. Consequently, these cell lines were used for further studies. Then, we treated SCC4 and SCC9 with two siRNA targeted to *TAB2*, and data showed that protein levels were greatly decreased (Figure 2(b)). The transfection experiments were optimized to minimize cytotoxicity. Cytotoxicity was determined by measuring the activity levels of the cells. Transfection experiments were optimized by treating OSCC cells with increasing amounts of siRNA and transfection reagents. The CCK-8 assay demonstrated that the downregulation of TAB2 inhibited cell proliferation dramatically (Figure 2(c)). Importantly, silencing of TAB2 promoted OSCC cell apoptosis (Figures 2(d) and 2(e)) and inhibited proliferative activity (Figures 2(f) and 2(g)). Thus, reduction of TAB2 expression could inhibit OSCC proliferation and induced apoptosis.

### 2.3. TAB2 Overexpression Promoted OSCC Cell Tumorigenicity

To further determine the function of TAB2 in OSCC, TAB2 was overexpressed in SCC1 cells. The efficiency of protein expression improvement was verified by western blotting assays (Figure 3(a)). As expected, TAB2 upregulation promoted cell proliferation according to the CCK-8 assay results (Figure 3(b)). Correspondingly, the flow cytometry captured lower rate of apoptotic cells (Figures 3(c) and 3(d)) and higher proliferation ability (Figures 3(e) and 3(f)) after extra acquisition of TAB2. Altogether, our data suggested that TAB2 might contribute to OSCC tumorigenicity.

### 2.4. TAB2 Regulates the PI3K-AKT Pathway and EMT Pathway in OSCC

To explore the underlying mechanism of how TAB2 in regulating OSCC progression, TCGA-HNSCC patients were divided into *TAB2* high expression and low expression groups for comparison and volcano scatter plot was used to separate the differentially expressed genes (DEGs) into up, not significant (not sig.), and downregulation genes (Figure 4(a)). Next, we performed gene ontology analysis using the up DEG data and found that increased mRNA in *TAB2* high expression group were enriched in epithelial-mesenchymal transition (EMT) and cell proliferation oncogenic pathways (Figure 4(b)). In addition, KEGG enrichment analysis results showed that up DEGs were enriched in oncogenic pathways including EMT and PI3K-AKT pathways (Figure 4(c)). To verify the results, expression of candidate genes was detected in protein level. First, apoptosis-related protein expression was upregulated in SCC9 when TAB2 was knockdown (Figure 4(d)), but it was downregulated in SCC1 cells when TAB2 was overexpressed (Figure 4(e)).

Downregulation of TAB2 decreased the participants of PI3K-AKT pathway and EMT pathway protein levels, including PI3K, AKT, SNAIL, and SLUG (Figure 4(f)). Similarly, overexpression of TAB2 could significantly increase the candidate genes expression (Figure 4(g)).

## 3. Discussion

It was anticipated that improved outcomes for patients with OSCC would result from developments in biotechnology, medication development, robotic surgery, radiation techniques, and molecular characterization of human malignancies. Nevertheless, despite these advancements, OSCC outcomes have largely stayed unchanged for the last few decades. This outcome is largely attributable to OSCC's extremely aggressive and metastatic character. A decisive factor in the multistage process of metastasis is the early step of local invasion of carcinoma cells [28–30]. However, the mechanisms coordinating the increased motility of proliferating cancer cells remain elusive. EMT is a widely known biological process that is essential to cancer progression [31, 32]. OSCC cells undergoing EMT exhibit downregulation of E-cadherin, upregulation of vimentin at the protein level, and reduced cell adhesion and enhanced migration and invasiveness at the cellular function level thereby promoting metastasis [33, 34]. The PI3K-AKT signaling pathway is an important cancer cell pathway. Among the signaling pathways that generally promote malignant transformation, the PI3K-AKT signaling pathway is the most frequently changed carcinogenic pathway in OSCC [35, 36]. Akt inactivates the proapoptotic factors Bad and procaspase-9 by phosphorylation to regulate apoptosis [37] and inhibits GSK3 to induce cell cycle progression via regulation of RB hyperphosphorylation and inactivation [38]. Akt also phosphorylates p21 and inhibits its antiproliferative effects by retaining it within the cytoplasm [39, 40].

Despite recent breakthroughs in current knowledge of the genetic and immunological profile of OSCC, there are still few clinically practical indicators. Therefore, specific therapeutic molecular targets for OSCC are urgently needed. In contrast, in our study, we demonstrated that TAB2 expression is specifically elevated in OSCC and correlates with clinical features. The value of expression of many molecules in predicting response to therapy, including immunotherapy, has not been previously demonstrated. However, high expression of TAB2 was associated with poor patient prognosis, demonstrating its potential as a molecular target. In addition, we found the function of TAB2 in promoting tumor progression in OSCC cell lines, and we creatively discovered the potential function of TAB2 in regulating EMT and PI3K-AKT pathways. Previous studies have shown that TAB2 play a necessary role in NF-kappaB pathway activation by binding to polyubiquitin chains [41, 42]. Importantly, the upregulation of the NF-kappaB signaling pathway in tumorigenesis has been confirmed [43–45], and the activation of NF-kappaB will upregulate the levels of EMT and PI3K-AKT pathway [46, 47] and promote tumor metastasis and proliferation. Intriguingly, our GO and KEGG analyses of TCGA data demonstrated that genes upregulated in the TAB2 high group are significantly associated with EMT and PI3K-AKT signaling pathway. Besides, we found that TAB2 deletion significantly downregulated the protein expression of key candidate genes in the EMT and PI3K-AKT pathways, while overexpression of TAB2 upregulated the protein expression, which also proved that TAB2 regulates the pathways. As thus, TAB2 is critical to the regulation of EMT and PI3K-AKT signaling pathways and may serve as a therapy target of tumor metastasis. At the same time, our results demonstrated that OSCC requires TAB2 for high proliferation and low apoptosis rate. Moreover, our patient cohort data showed that TAB2 was highly expressed in tumors and its expression was negatively correlated with overall survival. Thereby, our data provide a deeper understanding of TAB2 and new ideas for treatment in OSCC.

In conclusion, our study demonstrated that TAB2 is closely correlated with OSCC tumor progression. Mechanistically, we found the regulating role of TAB2 in EMT and PI3K-AKT pathways in OSCC. TAB2 can promote proliferation and inhibit apoptosis by regulating tumor-related pathways. From a clinical perspective, targeting TAB2 may be a promising strategy for OSCC. The current study does, however, have several drawbacks. The absence of experimental data from animal models that have been validated is a major limitation. More specialized experimental methods are required for verification of the mechanism. Although further research is needed to elucidate the carcinogenic mechanisms of TAB2 more fully, our current study lays the foundation for better treatment strategies.

## 4. Materials and Methods

### 4.1. Cell Culture

Human oral keratinocytes (HOK) were purchased from ScienCell (Carlsbad, California, USA). Oral squamous cancer cell lines (SCC1, HN6, SCC4, SCC9, and SCC15) were obtained from the American Type Culture Collection (ATCC; Manassas, USA). All the cells were maintained in Dulbecco's Modified Eagle's Medium (DMEM, 11885-076, Gibco, Waltham, USA) supplemented with 10% fetal bovine serum (FBS, 10270-106, Gibco) at a humidified incubator (5% CO_2_, 37°C). Mycoplasma testing on cell lines was performed frequently, and cultures of cell lines were limited to 20 passes.

### 4.2. Patient Specimens

In our study, 57 OSCC tissues and adjacent normal tissues were harvested from OSCC patients who underwent surgery in Hospital of Stomatology, Guanghua School of Stomatology, Sun Yat-sen University. Patients who received preoperative radiotherapy or chemotherapy were excluded. The overall survival (OS) time was from the date of diagnosis to September 2021 (or death). In the TAB2 expression study, 57 tumor samples and each corresponding nontumor tissue were collected from patients ranging in age from 42 to 85 years. All patients provided signed informed consents before enrollment. Our study was approved by the ethical committee of Shenzhen People's Hospital (No. LL-KY-2020054).

### 4.3. Cell Transfection

Small interference RNA (siRNA) transfection was conducted by Lipo 2000 transfection reagent (Thermo Fisher, Waltham, USA). TAB2 siRNA interference sequences are listed as follows: siTAB2-1: CAGCAUUAGUGAUGGACAAdTdT (sense) and UUGUCCAUCACUAAUGCUGdTdT (antisense) and siTAB2-2: GGUGCAUGUUACAGAAUAAdTdT (sense) and UUAUUCUGUAACAUGCACCdTdT (antisense).

The cytotoxicity of siRNA was tested using the CCK-8 kit (CCK-8, 500, Dojindo, Tokyo, Japan), which measures the activity of cells according to the manufacturer's protocol, with lower cellular activity indicating higher cytotoxicity.

In addition, plasmid expressing human TAB2 (Lv-TAB2) was used for overexpression of TAB2.

### 4.4. CCK-8 Assay

OSCC cell proliferative activity was measured via a cell counting kit-8 (Dojindo, Tokyo, Japan). Briefly, cells were seeded in 96-well plates (1 × 10^3^ per well) and incubated under 37°C. After adherence, the proliferation rates of cells were detected by the Infinite 200 PRO at indicated time points.

### 4.5. Cell Cycle Assay

OSCC cells were harvested 48 hours after transfection, followed by fixed overnight with ice-cold 75% ethanol and stained with the Cell Cycle kit (70-CCS012, MultiScience, Hangzhou, China) according to the standard protocol. Finally, cells were analyzed on a flow cytometry and CytExpert software.

### 4.6. Apoptosis Assay

Cell apoptosis rate was measured by the Annexin V Apoptosis Detection Kit (70-AP101-100, MultiScience) according to the standard protocol. In brief, OSCC cells were digested non-EDTA trypsin 48 hours after transfection and collected after discarding the supernatant. After staining the cells, fluorescence was detected on a flow cytometry and CytExpert software calculate cell apoptosis.

### 4.7. Western Blotting

OSCC cell protein was harvested by ice-cold RIPA lysis solution, and protein concentration was determined by the Pierce™ BCA Protein Assay Kit (Thermo Fisher Scientific, Waltham, USA). The protein was separated by SDS-polyacrylamide gel electrophoresis and then transferred to polyvinylidene fluoride (PVDF) membrane by wet transfer method. Finally, the protein bands were sequentially probed with primary and HRP-conjugated secondary antibodies, after which protein-antibody complex was visualized by enhanced chemiluminescence (ECL) reagent.

Antibodies for GAPDH (ab9485, Abcam, Cambridge, UK), SNAIL (ab216347, Abcam), and SLUG (ab51772, Abcam) were purchased from Abcam. Antibodies for TAB2 (14410-1-AP, Proteintech, Rosemont, USA), PI3K (20584-1-AP, Proteintech), and AKT (60203-2-Ig, Proteintech) were purchased from Proteintech. Antibodies for Caspase-3 (9662s, Cell Signaling Technology, Boston, USA), Caspase-8 (4790S, Cell Signaling Technology), Caspase-9 (9504S, Cell Signaling Technology) were purchased from Cell Signaling Technology.

### 4.8. Immunohistochemistry Staining

The OSCC sections were deparaffinized and rehydrated, and antigen was retrieved according to the standard protocol, followed by removing endogenous peroxidases. Then, sections were incubated with the primary antibodies at 4 °C overnight. Thereafter, HRP-labeled secondary antibodies were added for 1 hour at room temperature. 3,3′-Diaminobenzidine (AR1022, DAB, BOSTER, Wuhan, China) staining solution was utilized to develop the gene expression. IHC staining intensity scores were 0 (negative), 1 (weak), 2 (medium), and 3 (strong). IHC score was defined as multiplying the percentage of positive cells (P) by the intensity (I). The formula is as follows: *Q* = *P* × *I* and Maximum = 300.

### 4.9. TCGA Data

The gene expressions of 520 patients with HNSCC (head and neck squamous cell carcinoma) and 44 normal samples were obtained from The Cancer Genome Atlas (TCGA) database. In this study, we analyzed the mRNA expression levels of *TAB2* in HNSCC by UALCAN data (http://ualcan.path.uab.edu).

### 4.10. KEGG and Gene Ontology Analyses

To investigate the relationship between TAB2 and OSCC pathogenesis, KEGG and Gene Ontology analyses were conducted using DAVID Bioinformatics Resources 6.8 (https://david.ncifcrf.gov).

### 4.11. Statistical Analysis

Data was expressed as mean ± SD of at least three biological replicates. Results between two groups were compared by Student's *t*-tests. OS (overall survival) rate was compared based on the Kaplan-Meier method and paired with log-rank test. Analyses of all data were performed by GraphPad Prism 8.0 and *P* value < 0.05 was regarded to be statistically significant.

## Figures and Tables

**Figure 1:** TAB2 expression was upregulated and correlated with poor prognosis in OSCC. (a) Expression analysis of TAB2 in HNSCC tissue (*n* = 520) and normal tissue (*n* = 44) using TCGA database. (b) Box plots comparing the expression of TAB2 in different HNSCC tumor grade. (c) Representative IHC images of OSCC tissues (*n* = 57) to show the expression of TAB2 in tumors or corresponding normal tissues. Scale bar, 100 *μ*m. (d) The TAB2 IHC score quantification. (e) Effect of TAB2 expression level on OSCC patient overall survival (*n* = 45). Patients were divided into TAB2 high group and TAB2 low group according to the IHC results.

**Figure 2:** Deletion of TAB2 in OSCC cells displays decreased proliferation and increased apoptosis. (a) Western blot was used to detect TAB2 expression in six OSCC cell lines. (b) Confirmation of siRNA reduced TAB2 protein expression level by Western blot in SCC4 and SCC9 cell lines. (c) CCK-8 assay was used to detect the proliferation ability in SCC4 and SCC9 cells with TAB2 transient knockdown. (d and e) Inhibition of TAB2 could induce the apoptosis of SCC4 and SCC9 cells. (f and g) Knockdown of TAB2 results in the reduction of cell proliferation.

**Figure 3:** Overexpression of TAB2 promotes OSCC progression. (a) Overexpression of TAB2 in SCC1 cell line was verified by western blotting. (b) CCK-8 kit is utilized to determine the proliferation in SCC1 after TAB2 was overexpressed. (c and d) TAB2 contributes to the apoptosis inhibition in SCC1 cells. (e and f) TAB2 overexpression promotes the proliferation ability of SCC1 cells.

**Figure 4:** TCGA analysis reveals that TAB2 regulates EMT and PI3K-AKT pathway in OSCC. (a) Differentially expressed genes are shown by volcano scatter plots. Blue dots represent downregulated genes in TAB2 high expression group, gray represents no significant change genes, and red represents upregulated genes. (b) The Gene Ontology biological process enrichment analysis of DEGs identified the most relevant function modulated by TAB2. (c) The KEGG enrichment analysis was performed to obtain downstream signaling pathway by monitoring upregulated DEGs. (d and e) Western blot analysis of caspase-3, 8, and 9 genes in SCC9 and SCC1 cell lines. (f and g) Western blot analysis of EMT and PI3K-AKT pathway key genes using indicated antibodies in SCC9 and SCC1 cell lines.

## Data Availability

The datasets used and/or analyzed during the current study are available from the corresponding author on reasonable request.

## Abbreviations

DAB: 3,3′-Diaminobenzidine
DEGs: Differentially expressed genes
EMT: Epithelial-mesenchymal transition
GO: Gene Ontology
OS: Overall survival
TAB2: Transforming growth factor *β*-activated kinase 1 binding protein 2.
